The article "Nanohydroxyapatite-Blasted Bioactive Surface Drives Shear-Stressed Endothelial Cell Growth and Angiogenesis" was published in 2022. Journal: Biomed Res Int.

# Nanohydroxyapatite-Blasted Bioactive Surface Drives Shear-Stressed Endothelial Cell Growth and Angiogenesis

**DOI:** 10.1155/2022/1433221

**Published:** 2022-02-23

**Authors:** T. S. Pinto, B. R. Martins, M. R. Ferreira, F. Bezerra, W. F. Zambuzzi

**Affiliations:** Lab. of Bioassays and Cellular Dynamics, Department of Chemical and Biological Sciences, Institute of Biosciences, UNESP-São Paulo State University, 18618-970, Botucatu, São Paulo, Brazil

## Abstract

Nanosized crystalline hydroxyapatite coating (HAnano®) accelerates the osteointegration of dental implants which is hypothesized to drive angiogenesis. In order to test this hypothesis, we have subjected shear-stressed human umbilical vein endothelial cells (HUVECs) to a HAnano®-enriched medium, as well as to surface presenting dual acid etching (DAE) as a control. To note, the titanium implants were coated with 10 nm in diameter HA particles using the Promimic HAnano method. Our data reveals that HAnano® modulates higher expression of genes related with endothelial cell performance and viability, such as VEGF, eNOS, and AKT, and further angiogenesis in vitro by promoting endothelial cell migration. Additionally, the data shows a significant extracellular matrix (ECM) remodeling, and this finding seems developing a dual role in promoting the expression of VEGF and control endothelial cell growth during angiogenesis. Altogether, these data prompted us to further validate this phenomenon by exploring genes related with the control of cell cycle and in fact our data shows that HAnano® promotes higher expression of CDK4 gene, while p21 and p15 genes (suppressor genes) were significantly lower. In conjunction, our data shows for the first time that HAnano®-coated surfaces drive angiogenesis by stimulating a proliferative and migration phenotype of endothelial cells, and this finding opens novel comprehension about osseointegration mechanism considering nanosized hydroxyapatite coating dental implants.

## 1. Introduction

Advances in metallic based biomaterials were dynamically achieved over the last years and have proposed optimized materials in the biomedical field to replace or sustain a lost bone function [1]. There are many characteristics of metal implants that develop essential functions in the success of biomaterial biocompatibility and performance, and these issues affect several biological processes, such as endothelial cells (EC) and blood platelets, responsible for triggering signaling involved with local inflammation, blood coagulation, angiogenesis, and others [2]. Considering the osseointegration biology of dental implants, this is expected that the biology of the reactional tissue surround the implanted devices need to recapitulate principles of osteogenesis in an appositional bone growth manner by requiring a plethora performance of undifferentiated and osteogenic cells and also require specific intracellular pathways to drive the cell adhesion, proliferation, and differentiation [3, 4].

Although titanium alloys have been widely used in dentistry mainly considering their characteristics such as stability, mechanical strength, and corrosion resistance [5], there is constant interest in ameliorating their performance by proposing the most sophisticated surfaces considering more than physicochemical properties, applying the knowledge on the bioactive performance of coatings, as well as nanotechnology and how much these surfaces could be predicted considering the biological responses [6, 7]. As it has been related in other studies, a novel surface blasted with nanosized hydroxyapatite (0.02 *μ*m thin; HAnano®, Promimic, Gothenburg, Sweden) is proposed with already known biological responses [6, 7] mainly based on their superhydrophilic surface without changing the microstructure of the dental implants [8]. It is important to mention that HA is the major inorganic component of the bone, and it seems to favor the success of bone cell interaction and osteogenesis [9], and it seems HAnano® be a bioinspired surface.

Recently, we have focused on evaluating the relevance of intracellular signaling pathways in driving the interface of tissue with the implants [10–14], mainly considering the releasing debris/molecules from these materials and whether these materials could affect blood vessels and osteogenesis [15]. Additionally, this is known that the clinical success of the treatment using biomaterials depends on adequate blood apport to deliver important nutrients and biomolecules to the injured tissue during osseointegration and angiogenesis and seems develop a pivotal role maybe coupling osteoblast's differentiation and also enhancing bone healing [16].

Angiogenesis in bone tissue is crucial during development and healing and during its remodeling; it involves a critical interaction with bone cells preceding the onset of osteogenesis by activating a plethora of proangiogenic factors such as vascular endothelial growth factor (VEGF), platelet-derived growth factor (PDGF), transforming growth factor beta (TGF-*β*), fibroblast growth factors (FGF), and bone morphogenetic proteins (BMPs). In this way, Kusumbe et al. identified a new capillary subtype able to couple angiogenesis to osteogenesis by generating a distinct microenvironment and maintaining perivascular osteoprogenitors [17]. Importantly, these mechanisms seem to require a dynamic extracellular matrix (ECM) remodeling in response to biomaterials and this mechanism is devoted to the matrix metalloproteinase (MMP) activities [18].

Blood vessels play a pivotal role in bone development, remodeling, and homeostasis; its being in the angiogenesis is crucial during the bone healing surrounding the dental implants. In this way, although some progress has been achieved regarding the HAnano® promoting osteogenesis, very few is documented about angiogenesis in this aspect. Thus, we have hypothesized that HAnano® drives angiogenesis surrounding the implants and guarantees the success of its osseointegration when coating titanium-based dental implants. To better address this issue, we have subjected shear-stressed human umbilical vein endothelial cells (HUVECs) to HAnano®-enriched medium up to 24 hours when the biological samples were collected to allow further the molecular analysis. Importantly, the endothelial cells were maintained in vitro considering the shear stress mimicking blood tensional forces [19, 20]. Summarizing, our data shows clearly that HAnano® activates genes related with angiogenesis and promotes the proliferation/migration of endothelial cells by coordinating ECM remodeling and higher expression of genes related with endothelial cell growth and migration.

## 2. Material and Methods

### 2.1. Implants and Reagents

#### 2.1.1. Implants

The titanium-based dental implants evaluated in this study presenting DAE surfaces and EPIKUT® with HAnano® surface were obtained from S.I.N. Implant System, Sao Paulo, Brazil, with 3.5 mm in diameter and 10.0 mm in length. HAnano® surface was obtained using the Promimic HAnano method [21, 22]. Briefly, the samples were dipped into a stable particle suspension containing 10 nm in diameter HA particles followed by a heat treatment at 550°C for 5 min in a nitrogen atmosphere. Importantly, the calcium to phosphor ratio is 1.67. The surfactant-mediated process allows better control of the chemical composition of the coating [22], which has a thickness of less than or equal to 150 nm.

#### 2.1.2. Reagents

RPMI medium, fetal bovine serum (FBS), trypsin, penicillin, and streptomycin (antibiotics) were purchased from Nutricell (Campinas, Sao Paulo, Brazil). Trypan Blue (T6146), acetic acid glacial (695092), (3-(4,5-dimethylthiazol-2-yl)-2,5-diphenyltetrazolium bromide) (MTT) (M2128), ethanol (459844), and crystal violet dye (C0775) were purchased from Sigma Chemical Co. (St. Louis, MO, USA). TRIzol™ reagent (15596026), DNase I (18068015), and High-Capacity cDNA Reverse Transcription Kit (4368814) were obtained from Thermo Fisher Scientific Inc. (Waltham, Massachusetts, EUA). GoTaq qPCR Master Mix (A6002) was purchased from PROMEGA (Madison, Wisconsin, EUA). Oligonucleotides for gene expression, microRNA, and promoter methylation were purchased from Exxtend (Campinas, São Paulo, Brazil).

### 2.2. Cell Culture

In this study, the cell line used was human umbilical vein endothelial cells (HUVECs) (ATCC; CRL-1730; passage < 10). HUVECs were cultivated in RPMI medium (Nutricell, Campinas, Brazil) supplemented with penicillin (100 U/mL) and streptomycin (100 mg/mL) and 10% fetal bovine serum (FBS) and maintained at 37°C with 5% CO_2_. HUVECs were seeded in the peripheral area of the modified 100 mm culture dishes to allow the application of shear stress methodology. To note, the modified 100 mm culture dishes were obtained by bonding at the bottom a 60 mm culture dishes into their center using medical silicone, and thereafter, the dishes were sterilized using UV light for 30 min [20, 23–25] (Figure 1).

### 2.3. Shear Stress Model

HUVECs were previously seeded onto the peripheral area of the modified culture dishes (as described earlier) and then subjected to the orbital shear stress-induced tension force, using an orbital shaker (Scilogex, Rocky Hill, CT) positioned inside of the cell culture incubator, at 37°C in the presence of CO_2_ and 95% humidity, as proposed by others [19, 20, 23, 26–28]. The shear stress model performed here uses an orbital shaker respecting the formula of the maximal wall shear stress: *τ*max = *α*√*ρη*(2*πʄ*)3, in which *τ*max (Pascal unit) is the shear stress, *α* is the radius of orbital rotation (12 cm), *ρ* is the density of the cell culture medium (937.5 kg/m^3^), *η* is the viscosity of the cell culture medium (7.5 × 10^−4^ Pa s), and *ʄ* is the frequency of rotation. The titanium-enriched medium was used to treat monolayers of endothelial cells in this shear stress workflow in a rotation frequency of 100 rpm, respecting the protocol of previous studies, which is within the range of physiological arterial shear stress (~1–4 Pa). Thus, HUVECs remained in this workflow up to 24 h, being subjected to different treatments: HAnano®-enriched medium and dual acid-etched- (W/DAE-) enriched medium; both were compared to the control (when the cultures were maintained without any treatment). The samples of each group were properly collected to allow the molecular analysis, as schematized in Figure 1.

### 2.4. Conditioned Medium Obtention

To prepare the titanium-enriched medium, both dual acid-etching (DAE) treating surface (named W/DAE) and the nanohydroxyapatite-blasted surfaces (named HAnano®) were incubated in cell culture media (RPMI) without FBS up to 24 h at 37°C, 5% CO_2_, and 95% humidity (0.2 g/mL (*w*/*v*); ISO 10993:2016), as we have proposed earlier to evaluate biomaterials [11, 29, 30]. This is expected that the conditioned medium contains molecules released from those metallic alloys and might affect the biology of endothelial cells. The cytotoxic effect of those implants was measured using MTT assay.

### 2.5. Ti Amount Was Measured by Graphite Furnace Atomic Absorption Spectrometry

The conditioned medium was used to measure Ti element content before and after treating the HUVECs in the shear stress model. Importantly, Ti determination was performed by a graphite furnace atomic absorption spectrometry, in which the graphite tube's heating program optimized for Ti determinations was based on the procedure described by Silva et al. [31].

### 2.6. Cell Viability Assay

The conditioned medium was prepared using the ISO 10993:2016, as well as it has been used by Zambuzzi et al. [32]. To prepare the conditioned medium, the implants were incubated in RPMI up to 24 hours. Previously, the cells were seeded on 96-well plates (5 × 10^4^ cells/mL) and incubated up to 24 h with the conditioned medium, when the culture media was substituted by 180 *μ*L/well of each sample extract plus 20 *μ*L FBS (resulting a final concentration of 10% of FBS). The control cultures were considered maintaining cells under classical cell culture conditions. The experimental time was 24 hours, when the cell viability was assessed by adding 1 mg/mL of 3-(4,5-dimethyl-2-thiazolyl)-2,5-diphenyl-2H-tetrazolium bromide (MTT) to measure the mitochondrial dehydrogenase activity by MTT reduction up to 3 hours into CO_2_ incubator, where there is a conversion of the yellow water-soluble tetrazolium salt MTT into the purple-colored soluble compound of formazan. The formazan was solubilized into ethanol, and the absorbance measured at 570 nm (Synergy II; BioTek Instruments, USA).

### 2.7. Cell Adhesion Assay

For evaluating cell adhesion performance, endothelial cells were trypsinized, properly counted, and then reseeded (1 × 10^4^ cells per well) in sextuplicate into 96-well plates in implant-conditioned medium supplemented with 10% of FBS and 1% antibiotics up to 24 h. Then, the nonadherent cells were removed by washing with PBS (37°C) and the adherent cells fixed in glacial acetic acid and absolute ethanol solution (3 : 1; *v*/*v*) for 10 minutes at room temperature (RT). Thereafter, the cells were stained with 0.1% (*w*/*v*) crystal violet for 10 minutes at RT. The excess dye was retained by decanting and washing (2x) with distilled water. Finally, the dye was extracted with 10% acetic acid (*v*/*v*) and the optical density measured at 550 nm using a microplate reader (Biotek Co., Winooski, VT). For the positive control, the cells were seeded on polystyrene surface (control group (Ctrl)). The results were expressed as percent of the control (100%).

### 2.8. Angiogenesis Assay

The cell migration and angiogenesis were estimated by using a scratch assay, as performed earlier [19]. The scratch assay estimates the cell migration and angiogenesis. Briefly, the cells were cultured in 12-well plates at 4 × 10^4^ cells/cm^2^, and after 100% confluence, an introduced area was cleared using a pipet tip [19] and then a monitoring of the angiogenesis and the migration of the ECs up to 12 h and 16 h. Thereafter, the cultures were subjected to fixation with 4% PFA and stained with Alizarin Red S. In the analysis of the angiogenesis in vitro, the wound healing area was measured in an inverted microscope with a coupled digital camera (Zeiss) and the acquired images analyzed using the ImageJ software (NIH, Bethesda, MD).

### 2.9. Total mRNA Isolation and RT-qPCR Analysis

In order to evaluate the molecular behavior of genes related with angiogenesis and cellular survival in response to HAnano®, the cells were newly subjected to the conditioned medium containing the released molecules and further harvested and total mRNA properly isolated using Ambion TRIzol Reagent (Life Sciences, Thermo Fisher Scientific Inc., Waltham, MA) and treated with DNase I (Invitrogen, Carlsbad, CA). Complementary DNA (cDNA) synthesis was performed with the High-Capacity cDNA Reverse Transcription Kit (Applied Biosystems, Foster City, CA) according to the manufacturer's instructions. Real-Time Reverse Transcriptase qPCR was carried out in a total of 10 *μ*L, containing PowerUp™ SYBR™ Green Master Mix 2× (5 *μ*L; Applied Biosystems, Foster City, CA), 0.4 *μ*M of each primer, 50 ng of cDNA, and nuclease-free H_2_O. Results were expressed as relative amounts of the transcripts using 18s as reference gene (housekeeping gene), using the cycle threshold (Ct) method. Primers and work conditions are described in Table 1.

### 2.10. Statistical Analyses

Results were represented as mean ± standard deviation (SD). The samples assumed a normal distribution, and they were subjected to Student's *t*-test (two-tailed) with *p* < 0.05 considered statistically significant. In the experiment where there were more than two groups, we used one-way ANOVA with Tukey's multiple comparisons test, in order to compare all pairs of groups. In this case, the significance level was considered when alpha = 0.05 (95% confidence interval). The software used was GraphPad Prism 7 (GraphPad Software, USA).

## 3. Results

Firstly, we have focused on evaluating whether the different surfaces of titanium proposed in this study were able to develop some cytotoxicity in endothelial cells. Thus, Figure 2(a) shows that there is no significance effect on mitochondrial activities in response to both surfaces, as well as the cell adhesion, once Figure 2(b) brings the same behavior of endothelial cells responding to the materials, without any changes on the outcomes obtained by shear-stressed endothelial cells. Additionally, we have also investigated whether endothelial cells were able to capture titanium released from the materials, and our data shows for the first time there is a significant uptake of titanium by shear-stressed endothelial cells responding to HAnano® super hydrophilic surface (Figure 2(c)) and this data could explain some metabolic changes in those cells.

Thereafter, in order to investigate whether the Ti-enriched medium was able to change the metabolism of shear-stressed endothelial cells, we evaluated genes related with endothelial cells phenotype: importantly, our data shows that shear-stressed endothelial cells responding to HAnano® super hydrophilic surface presents a significant higher expression profile of VEGF (Figure 3(a); about 10-fold changes), eNOS (Figure 3(b); about 4-fold changes), and AKT (Figure 3(c); about 2.5-fold changes).

In addition, this data prompted us to better evaluate the behavior of shear-stressed endothelial cells by considering a well-accepted in vitro methodology. In general, shear-stressed endothelial cells responding to Ti-enriched medium presented a better performance in cell migration and angiogenesis in vitro than control cultures (Figures 4(a)–4(j)), with better outcomes obtained in response to HAnano® superhydrophilic surface in 16 hours (Figure 4). Figure 4(k) brings the analysis of the wounding area; considered here, the capacity of endothelial cells migrate responding to the specific treatments.

As migration and proliferation actions of the cells requires a dynamic mechanism of extracellular matrix (ECM) remodeling, we also investigated the behavior of matrix metalloproteinase (MMP) activities, and our data supports that shear-stressed endothelial cells responding to the Ti-enriched medium promoted a higher activity of MMP2 (Figures 5(a)–5(d)). Here, we need to consider the limitation of the experimental model used in this study, and the data supports a significant stimulus of Ti-enriched medium on remodeling ECM in endothelial cells.

To better understand the behavior of shear-stressed endothelial cells responding to Ti-enriched medium obtained by surfaces DAE and HAnano®, we now investigated the relevance of genes related with cell proliferation. Our data shows there is a significant downregulation of genes of MAPKs p38 and ERK in endothelial cells responding to Ti-enriched medium, and it does not matter the kind of surface evaluated (Figures 6(a) and 6(b)). In addition, specific genes related with cell cycle progression were also investigated and Figure 6(c) shows there is a significant higher expression of CDK4 gene by shear stressed endothelial cells responding to HAnano® super hydrophilic surface, while CDK2 gene was significant downregulated (Figure 6(d)). These data could explain the findings shown previously here in cell migration and angiogenesis in response to HAnano® surfaces. Importantly, in this context and considering the regulation of cell cycle activity of endothelial cells, we also investigated the behavior of genes related to negatively control cell proliferation, p15 and p21, and our data shows there is a significant downregulation of the expression profile of these both genes in endothelial cells responding to Ti-enriched medium, mainly considering p21 gene in response to HAnano® (Figures 6(e) and 6(f)).

## 4. Discussion

Considering the osseointegration-related microenvironment, angiogenesis is an important biological event to be considered, which plays a pivotal role on supplying cells, nutrients, and gases changes as well as clearing up waste molecules from the cellular metabolism. In addition, the vascularization plays crucial role in bone healing, mainly considering the coupling mechanism between bone cells and endothelial cells by angiocrine signals addressing bone cell activities and further osteogenesis. Once angiogenesis in response to biomaterials is barely understood, we decided to better evaluate the behavior of shear-stressed endothelial cells responding to Ti-enriched medium obtained from 2 different types of modified surfaces, as follows: (1) subjected to DAE (w/DAE) and (2) DAE-modified surfaces coated with nanosized HA (HAnano®). It is important to mention that we have previously shown that HAnano® superhydrophilic surface drives osteoblast performance when modifying dental implants surfaces [33].

In this study, our data shows that dental implants having HAnano® superhydrophilic surfaces generates an adequate microenvironment to drive angiogenesis and this study could explain the success of its clinical application [34]. Firstly, our data shows that shear-stressed endothelial cells significantly uptake titanium released from HAnano®-enriched medium and this data opened a set of question about the behavior of endothelial cells and angiogenesis and, in part, is shown here. Importantly, our data shows that conditioned medium by HAnano® promotes higher expression of important genes related with endothelial cell phenotype: VEGF and eNOS. Importantly, these data bring important evidences to suggest the relevance of angiogenesis during tissue remodeling microenvironment surrounding the dental implants. This is known that angiogenesis is regulated by many growth factors and molecules, and in this scenario, VEGF and nitric oxide (NO) are potent angiogenic factors.

Mechanistically, the capacity of VEGF in promoting bone regeneration and healing has been shown in several biological models [35–37]. VEGF is a very important growth factor in the vascular system driving endothelial cell growth and survival, as well as develops a signaling hub with osteogenesis by regulating the expression of bone morphogenetic proteins (BMPs) [38, 39], and VEGF may be released during matrix remodeling orchestrated by MMP-mediated matrix breakdown, which induces vascular invasion and angiogenesis [40]. Importantly, we have shown previously that titanium-based devices drive matrix remodeling by upmodulating the activities of matrix metalloproteinases (MMPs) [6, 29, 41] and this recapitulates events are also shown in bone development and healing [27, 42–47]. Importantly, this could be a prerequisite also to favor the angiogenesis process throughout the distraction osteogenesis phase, but to a lesser extent during the phase of consolidation [48], respecting distinct phases of bone repair progress.

Another concern evaluated here was the possibility of shear-stressed endothelial cells in expressing eNOS in response to nanosized HA, once the role of the messenger molecule nitric oxide has been evaluated in fracture healing [49], and NO is synthesized by three kinds of nitric oxide synthase (NOS): inducible NOS (iNOS), endothelial (eNOS), and neuronal (nNOS). Regarding eNOS, our data show a very similar profile of VEGF and seems to develop a pivotal role in endothelial cell activity to maintain endothelial homeostasis during bone healing surrounding the implanted devices. As we have also noticed from the data, a higher expression of AKT gene in endothelial cells responds to HAnano®; this seems obvious suggesting that the angiogenic stimulus of HAnano® requires AKT/eNOS axis in shear-stressed endothelial cells; once, this is widely related in the literature that AKT activates eNOS via activation of mTOR [50, 51]. Thus, AKT is closely linked to the formation of new blood vessels through the activation of endothelial nitric oxide synthase (eNOS) [52], which is responsible for relaxing vascular smooth muscle and also mediates angiogenesis by controlling the action of VEGF [52–54]. Moreover, Akt also regulates PI3K-mediated cell survival and is sufficient to block cell death induced by a variety of apoptotic stimuli [55, 56] and the importance of PI3K in endothelial cell was shown by using wortmannin as an inhibitor [28].

Finally, we have also investigated whether these molecular mechanisms led to the proliferation and migration of endothelial cells. Thus, we have further investigated angiogenesis in vitro by using a well-accepted functional assay and our data validates this hypothesis; once, endothelial cells subjected to HAnano® presented better cell cycle performance by upmodulating CDK4 gene and ECM remodeling, while both investigated cell cycle suppressor genes p15 and p21 were downmodulated. ECM remodeling seems to be an important hub in endothelial cells responding to HAnano® by favoring as a prerequisite to VEGF expression and also related with the growth of cells during angiogenesis. Generally, this is reasonable to suggest that HAnano® promotes an ideal microenvironment for osseointegration by regulating genes related with endothelial cell growth, such as VEGF, which could play an autrocrine loop and AKT/eNOS signaling, culminating with EC proliferation and angiogenesis, which could be coupled to osteogenesis; once, we have shown earlier the osteogenic effect of HAnano®.

In conjunction, this study brings sufficient in vitro data to support the angiogenic effect of HAnano®-coated titanium surface by modulating the proliferative and migration phenotype of endothelial cells, and these data partially explain a better performance of the application of HAnano® in vivo [34], maybe by coupling angiogenesis and osteogenesis during its osseointegration processes.

## Figures and Tables

**Figure 1:** Experimental design of this study. In order to evaluate the endothelial cell (EC) behavior in response to HAnano®, the conditioned medium was obtained in according to ISO 10993:2016 and further used to treat the endothelial cells for 24 h in an in vitro mimicking shear stress model, when the samples were properly collected to allow the molecular analysis.

**Figure 2:** HAnano® cytotoxicity and the capacity of shear-stressed endothelial cell in capturing medium-soluble titanium. The titanium-enriched medium was obtained in according to ISO 10993:2016 by incubating the implants containing DAE (w/DAE) or nanosized hydroxyapatite (HAnano®) coatings up to 24 hours and thereafter used to subject endothelial cell. Our data shows there is no effect on endothelial cell viability (a) and endothelial cell adhesion (b). Additionally, it was confirmed that shear-stressed endothelial cell captures a significant amount of medium-soluble titanium mainly responding to HAnano®. A significant difference was considered when *p* < 0.05.

**Figure 3:** HAnano® upmodulates EC phenotype-related genes. Shear-stressed endothelial cell were subjected to Ti-enriched medium for 24 hours, and the samples were harvested to allow gene expression using RT-qPCR methodology. Our data shows there is a significant higher expression of VEGF (a) and eNOS (b) genes in response to HAnano®, as well as AKT gene (c). The graphs bring the *n*-fold change of the profile of transcripts normalized to the 18S gene (housekeeping gene). Significant differences were considered when *p* < 0.05, represented by ^∗^ when compared to the Ctrl group and by ^#^ when compared to the W/DAE group.

**Figure 4:** The angiogenic effect of HAnano® was measured by a wound healing assay. (a) Endothelial cell forming a confluent monolayer. (b) In vitro “wound” was created by a straight-line scratch across the endothelial cell monolayer (*T*0). At time 0 (*T*0), the endothelial cell were scratched and subjected to conditioned medium, respecting the culture groups, as follows: Ctrl: RPMI (c, g); shear stress: endothelial cell in shear stress model (d, h); shear stress W/DAE: shear-stressed endothelial cell subjected with Ti-enriched medium by DAE (w/DAE) (e,i); shear stress HAnano®: shear-stressed endothelial cell subjected with Ti-enriched medium by HAnano® (nano-HA) (f, j). The scratch wound assay was used to assess the migration capacity of the endothelial cells under different conditioned media. The wound area was estimated by calculating the cell-free area in captured images using the ImageJ software (NIH, Bethesda, MD). The migration rate is expressed in percentage as the change in the wound area over time, the scratch area at time point 0 hours was set to 100%, and the other ones are represented as wound closure expressed as the remaining area uncovered by the cells in percentage. (k) The statistically significant changes are represented by ^∗^ when compared with the Ctrl group, by ^@^ when compared to the SS group, and by ^#^ when compared to the W/DAE SS group. Significant differences were considered when *p* < 0.05.

**Figure 5:** Both Ti-related surfaces with DAE or HAnano® promote higher activity of MMP2 enzyme. The ECM remodeling was evaluated by checking the activities of MMPs in response to titanium-enriched media indirectly obtained by 2 different surfaces DAE (w/DAE) and nanohydroxyapatite-blasted titanium surface (HAnano®) applying zymography technology (a). MMP2 activity showed different activities profiles, mainly observed higher in response to both treatments when compared to Ctrl (b–d). Differences were considered significant when *p* < 0.05, represented by ^∗^ when compared with the Ctrl group. MMP: matrix metalloproteinase.

**Figure 6:** CDK4 is upmodulated in response to HAnano®. Thereafter, understanding its relevance on endothelial cells migration and angiogenesis, we postulated the hypothesis that HAnano® modulates cell cycle-related genes. Although MAPKs p38 (a) and ERK (b) genes were downregulated in response to HAnano®, CDK4 gene expression was significantly higher ((c) approximately 2.5-fold changes), while CDK2 gene was downregulated (d). Importantly, cell cycle suppressor genes, p15 (e) and p21 (f), were downregulated in response to both W/DAE and HAnano®. The graphs bring the *n*-fold change of the profile of transcripts normalized to the 18S gene (housekeeping gene). Significant differences were considered when p <0.05, represented by ^∗^ when compared with the Ctrl group and by ^#^ when compared to the W/DAE group.

**Table 1:** Expression *primers* sequences and qPCR cycle conditions.

Gene	Primer	5′-3′ sequence	Work condition
AKT	Forward 1	CAGCGCGGCCCGAAGGAC	95°C -3 s, 55°C -8 s, 72°C -20s
	Forward 2	GGACTCCCGTTTGCGCCAGT	
	Reverse	GACGCTCACGCGCTCCTCTC	
CFL1	Forward	TGTGCGGCTCCTACTAAACG	95°C -3 s, 55°C -8 s, 72°C -20s
	Reverse	TCCTTGACCTCCTCGTAGCA	
P15	Forward	GGGACTAGTGGAGAAGGTGC	95°C -3 s, 55°C -8 s, 72°C -20s
	Reverse	CATCATCATGACCTGGATCGC	
P21	Forward	GCTGCCGAAGTCAGTTCCTT	95°C -3 s, 55°C -8 s, 72°C -20s
	Reverse	ATCTGTCATGCTGGTCTGCC	
CDK2	Forward	CTTTGCTGAGATGGTGACTCG	95°C -3 s, 55°C -8 s, 72°C -20s
	Reverse	GCCTCCCAGATTCCTCATGC	
CDK4	Forward	CTCTCTAGCTTGCGGCCTG	95°C -3 s, 55°C -8 s, 72°C -20s
	Reverse	GCAGGGATACATCTCGAGGC	
VEGF	Forward	TGCAGATTATGCGGATCAAACC	95°C -3 s, 55°C -8 s, 72°C -20s
	Reverse	TGCATTCACATTTGTTGTGCTGTAG	
ENOS	Forward	TATTTGATGCTCGGGACTGC	95°C -3 s, 55°C -8 s, 72°C -20s
	Reverse	AAGATTGCCTCGGTTTGTTG	
P38	Forward	GAGAACTGCGGTTACTTA	95°C -3 s, 55°C -8 s, 72°C -20s
	Reverse	ATGGGTCACCAGATACACAT	
ERK	Forward 1	AACAGGCTCTGGCCCACCCAT	95°C -3 s, 55°C -8 s, 72°C -20s
	Forward 2	CGCCCCTCCAAACGGCTCAA	
	Reverse	GCAGCGCCTCCCTTGCTAGA	
ITGB1	Forward	GCCGCGCGGAAAAGATGAA	95°C -3 s, 55°C -8 s, 72°C -20s
	Reverse	TGCTGTTCCTTTGCTACGGT	
FAK	Forward	TCAGCTCAGCACAATCCTGG	95°C -3 s, 55°C -8 s, 72°C -20s
	Reverse	CTGAAGCTTGACACCCTCGT	
SRC	Forward	CAACACAGAGGGAGACTGGT	95°C -3 s, 55°C -8 s, 72°C -20s
	Reverse	AGCTTCTTCATGACCTGGGC	
18S	Forward	CGGACAGGATTGACAGATTGATAGC	95°C -3 s, 55°C -8 s, 72°C -20s
	Reverse	TGCCAGAGTCTCGTTCGTTATCG	

## Data Availability

The data that support the findings of this study are available from the corresponding author upon reasonable request.
